# Effect of Mobile Internet on Attitude and Self-Efficacy of Patients with Coronary Heart Disease Diagnosed by 12-Lead Holter ECG

**DOI:** 10.1155/2022/3414178

**Published:** 2022-01-07

**Authors:** Haitao Sun, Jing Li, Yue Wang, Xiaoke Ma

**Affiliations:** ^1^Department of Electrocardiogram Room, Yantai Yuhuangding Hospital Affiliated To Qingdao University, Yantai 264000, Shandong, China; ^2^Department of Electrocardiogram Room, Yantai City Hospital of Traditional Chinese Medicine, Yantai, Shandong, China

## Abstract

**Objective:**

To explore the effect of mobile Internet on attitude and self-efficacy of patients with coronary heart disease (CHD) diagnosed by 12-lead Holter ECG.

**Methods:**

The clinical data of 62 patients with CHD who underwent routine ECG examination (control group I) and 12-lead dynamic electrocardiogram (control group II) in our hospital (June 2017–December 2020) were retrospectively analyzed, and the clinical data of another 62 patients with CHD who received 12-lead Holter ECG examination combined with mobile Internet in our hospital at the same time (study group) were retrospectively analyzed. The clinical observation indexes of the three groups were compared.

**Results:**

No obvious difference in general data among groups (*P* > 0.05). Compared with the control group I, the positive detection rate (PDR) of the study group and the control group II was obviously higher (*P* < 0.05), and the PDR of the study group was obviously higher than that of the control group II, without remarkable difference between both groups (*P* > 0.05). Compared with the control group, the scores of CAS-R of the study group were obviously higher (*P* < 0.05), and self-efficacy of daily life, health behaviors, medication compliance, and compliance behavior of the study group was obviously better (*P* < 0.05). The diagnostic efficacy was derived by ROC curve analysis, 12-lead Holter ECG combined with mobile Internet + routine ECG > 12-lead Holter ECG combined with mobile Internet > 12-lead Holter ECG > routine ECG.

**Conclusion:**

Compared with the routine ECG, the sensitivity of 12-lead Holter ECG in the diagnosis of CHD is conspicuously higher. Meanwhile, 12-lead Holter ECG combined with mobile Internet can enhance the diagnostic efficiency and improve patients' perceived control attitude and self-efficacy.

## 1. Introduction

As a common type of heart disease, coronary heart disease (CHD) is a kind of atherosclerotic heart disease. In recent years, with the continuous improvement of people's living standards, the incidence of CHD is on the rise. For a long time, the basic principle of “early detection and early treatment” has always been advocated in clinical practice [1–3]. Routine ECG is the most common and convenient method for the diagnosis of the disease in clinic, especially for patients with acute attack, but it has limitations in initial screening and dynamic evaluation of prognosis, which is difficult to popularize [4–6], while the 12-lead Holter ECG can continuously record and analyze the changes of ECG of the patients in both active and quiet states for a long time, with more advantages of large amount of information and long recording time than the routine ECG. In addition, the 12-lead Holter ECG is more practical, easy, safe, and economical, which should be promoted [7–9]. In addition, the author's clinical experience found that self-efficacy and perceived control attitude are very important in the self-management of patients with CHD. To improve the diagnosis and management efficiency, our hospital combined 12-lead Holter ECG with mobile Internet, which greatly improved the treatment efficiency of patients. Few relevant studies are observed in China. Based on the above, this paper will explore the effect of mobile Internet on attitude and self-efficacy of patients with CHD diagnosed by 12-lead Holter ECG, and the results are as follows.

## 2. Methods

### 2.1. Screening and Grouping of Patients

The clinical data of 62 patients with CHD who underwent routine ECG examination (control group I) and 12-lead dynamic electrocardiogram (control group II) in our hospital (June 2017–December 2020) were retrospectively analyzed, and the clinical data of another 62 patients with CHD who received 12-lead Holter ECG examination combined with mobile Internet in our hospital at the same time (study group) were retrospectively analyzed. The clinical observation indexes of the three groups were compared. The study was approved by the Hospital Ethics Committee.

### 2.2. Inclusion Criteria

1. All patients were diagnosed as CHD by coronary angiography
2. Patients were ≥55 years old
3. No ST-T changes were found in ECG
4. Patients were diagnosed for the first time
5. Patients could make clear compliant
6. With complete medical records, patients and their families understood the study and signed the consent form

### 2.3. Exclusion Criteria

1. Patients suffered from frequent premature beats or severe arrhythmias
2. Patients were complicated with myocarditis, cardiac hypertrophy, or malignant tumors
3. Patients had a history or potential risk of myocardial infarction
4. Patients had severe liver and kidney dysfunction
5. Patients had potential factors causing ST changes in ECG
6. Patients had cognitive disorders or low compliance

### 2.4. Methods

Patients of the control group relaxed and took the supine position in a calm state. The patients received the routine ECG examination. Continuous tracings were then performed by using a 12-lead electrocardiograph (manufacturer: Biomedical Instruments Co., Ltd.), with the paper speed of 25 mm/s and the amplitude of 10 mm/mV to ensure the smooth and clear baseline of the recording paper. Then, the patients were examined by a 12-lead Holter ECG and were continuously monitored for 24 hours [10–13]. Finally, the information was processed, the follow-up was carried out, and the manual judgment and correction were performed. Then, the comprehensive diagnosis was carried out combined with patients' cognition and symptoms within 24 h.

The study group was examined by 12-lead Holter ECG examination combined with mobile Internet. The receiving doctor first transmited the patients' real-time vital sign information (12-lead Holter ECG, noninvasive blood pressure, blood oxygen saturation, and respiration) to the database of the Chest Pain Center (CPC) on WeChat, and the treatment team of CPC formulated an emergency plan based on the above information, mainly including the stability of the patients' vital signs, the loading dose of aspirin and clopidogrel, necessary sedation and analgesia, and cognitive intervention and behavioral intervention via the mobile phone.

### 2.5. Observation Indexes

The general data including age, course of disease, BMI, gender, hypertension, hyperlipidemia, hyperglycemia, high cholesterol, and education degree were counted.

Selective multiposition coronary angiography was performed with puncture of the right femoral or radial artery by Judkins method [14]. It indicated positive when at least one main coronary artery or its branches of diameter stenosis was ≥50%. The positive detection rates of routine ECG, 12-lead Holter ECG, and 12-lead Holter ECG with mobile Internet were observed and analyzed.

The Control Attitude Scale-Revised (CAS-R) [15] was used to evaluate the patients' perceived control attitude. The scale contained 8 items, with a total score of 40 points and by 5-level scoring method for each item. The higher the score, the better the patients' perceived control attitude. The retest reliability, split-half reliability, and Cronbach's *α* coefficient of the scale were, respectively, 0.825, 0.512, and 0.874.

The self-efficacy of patients was evaluated with reference to the Self-Efficacy Evaluation Scale for Patients with Coronary Heart Disease adapted by Kärner et al. [16]. The scale included four major aspects, daily life (diet control, diet structure, and exercise), health behavior (quitting smoking and drinking), medication compliance (persistent medication, timely medication, and medication conforming to dosage), and compliance behavior (monitoring of blood pressure, blood sugar and blood fat, regular follow-up, and mood control), with 10 items in total and each item for 5 grades (totally can, usually can, basically can, usually cannot, and totally cannot) scored as 4-0 points, respectively. The higher the score, the better the patients' self-efficacy. “Basically can” of each item was regarded as the baseline for achieving self-efficacy. The retest reliability, split-half reliability, and Cronbach's *α* coefficient of the scale were, respectively, 0.928, 0.954, and 0.948.

### 2.6. Statistical Processing

All statistical data of the study were processed by SPSS 22.0 to calculate the difference between groups, and the pictures were graphed by GraphPad Prism 7 (GraphPad Software, San Diego, USA). Including enumeration data and measurement data in the form of (*n* (%)) and (*x* ± *s*), respectively, the study used *x*^2^ test and *t*-test. The differences were statistically significant at *P* < 0.05.

## 3. Results

### 3.1. General Data

After statistical analysis, *P* > 0.05 was derived from the general data of the two groups, which met the study criteria for controlled experiments, see Table 1.

### 3.2. Positive Detection Rate

Compared with the control group I, the positive detection rate (PDR) of the study group and the control group II was obviously higher (*P* < 0.05), and the PDR of the study group was obviously higher than that of the control group II, without remarkable difference among groups (*P* > 0.05), see Figure 1.

### 3.3. Perceived Control Attitude

Compared with the control group, the scores of CAS-R of the study group were obviously higher (*P* < 0.05), and the difference between groups was statistically significant, see Figure 2.

### 3.4. Self-Efficacy

Compared with the control group, self-efficacy of daily life, health behaviors, medication compliance, and compliance behavior of the study group was obviously better (*P* < 0.05), see Table 2.

### 3.5. Diagnostic Efficacy

The diagnostic efficacy was derived by ROC curve analysis, 12-lead Holter ECG combined with mobile Internet + routine ECG > 12-lead Holter ECG combined with mobile Internet > 12-lead Holter ECG > routine ECG, see Figure 3 and Table 3.

## 4. Discussion

At present, coronary angiography is taken as the gold standard for the diagnosis of CHD, but the method is high-cost and invasive examination limited by equipment and technical conditions, which is difficult to popularize [6, 17–19]. Routine ECG is the simplest and most effective noninvasive examination for the diagnosis of CHD, and its diagnostic value has also been affirmed by the medical community. However, in recent years, a number of related studies have shown that angina pectoris caused by myocardial ischemia may not present with ischemic ST changes. Meanwhile, according to the investigation, about 30% of patients with chronic angina pectoris are diagnosed as normal at rest by ECG, which shows that the routine ECG has certain limitations in the diagnosis of CHD, with high rate of clinical missed diagnosis [20–22]. 12-lead Holter ECG has the function of 24 h automatic monitoring and comprehensive visualization of patients' condition of myocardial ischemia and can also analyze the condition by 24 h graph, trend graph, full view graph, and heart rate change graph, more closely monitoring the patients' condition and progress. To further improve patients' self-efficacy and attitude control, this study combined 12-lead Holter ECG effectively with mobile Internet and analyzed and summarized the effect on the positive detection rate of CHD by routine ECG, 12-lead Holter ECG, and 12-lead Holter ECG with mobile Internet. It was found that, compared with the control group I, the PDR of the study group and the control group II was obviously higher (*P* < 0.05), and the PDR of the study group was obviously higher than that of the control group II, without remarkable difference between both groups (*P* > 0.05). The results were consistent with the study of NAULT [23], indicating that the sensitivity of 12-lead Holter ECG was obviously higher than that of routine ECG, and 12-lead Holter ECG with mobile Internet could better improve PDR of CHD compared with 12-lead Holter ECG alone, but the difference was not remarkable, which may be due to small sample size.

The research of Ollila et al. [24] shows that early prevention, early diagnosis, and early treatment of CHD are vital to the quality of life and long-term survival rate of patients. However, with a long course of disease, CHD is easy to repeat and has strict requirements on lifestyle. Various factors are easy to lead to poor compliance behavior. Health risk factors mainly impact on the incidence and mortality of diseases from biological, psychological, and social aspects, which are changeable by intervention measures and measureable. Self-efficacy is the belief that determines whether a person can achieve the set goal, and improving self-efficacy is more conducive to promoting behavior change. The application and potential of self-efficacy in chronic disease management are to improve patient-centered compliance behavior and further improve patients' lifestyle and health. The results showed that compared with the control group, self-efficacy of daily life, health behaviors, medication compliance, and compliance behavior of the study group was obviously better (*P* < 0.05), which indicated that self-efficacy suggested the formation and maintenance mechanism of human behavior from a new perspective, and self-efficacy level was a strong predictor of behavior implementation and change. The results suggested that 12-lead Holter ECG with mobile Internet was more conducive to the improvement of self-efficacy in patients with CHD. In addition, compared with the control group, the scores of CAS-R of the study group were obviously higher (*P* < 0.05), suggesting that the 12-lead Holter ECG with mobile Internet could effectively improve the health behaviors, perceived control attitude, and mood state. It was mainly because 12-lead Holter ECG based on mobile Internet greatly improved the diagnosis and treatment efficiency of patients, and the dynamic real-time data change was more capable of intuitively stimulating patients and improving their self-management efficacy and attitude control. Finally, the diagnostic efficacy was derived by ROC curve analysis, 12-lead Holter ECG combined with mobile Internet + routine ECG > 12-lead Holter ECG combined with mobile Internet > 12-lead Holter ECG > routine ECG, which demonstrated that 12-lead Holter ECG had absolute advantages in CHD diagnosis, and it combined with routine ECG could better improve the diagnostic efficacy.

To sum up, compared with the routine ECG, the sensitivity of 12-lead Holter ECG in the diagnosis of CHD is conspicuously higher. Meanwhile, 12-lead Holter ECG combined with mobile Internet can enhance the diagnostic efficiency and improve patients' attitude and self-efficacy. However, the sample size of this study is small, and it is still necessary to expand the sample for further exploration of comparative diagnosis accuracy. Moreover, mobile Internet is in need of further upgrading in practical application. In the development and application of WeChat database, it should not only combine with the characteristics of CHD but also refer to other basic diseases such as diabetes and hypertension.

## Figures and Tables

**Figure 1:** PDR of patients (%). Note: the abscissa indicates groups, and the ordinate indicates the percentage. The PDR of the control group I was 29 (46.77%). The PDR of the control group II was 55 (88.71%). The PDR of the study group was 57 (91.94%). ^*∗*^indicates the obvious difference in PDR between the control group I and the control group II (*X*^2^ = 24.948, *P* < 0.001). ^*∗∗*^indicates the obvious difference in PDR between the control group I and the study group (*X*^2^ = 29.748, *P* < 0.001).

**Figure 2:** Scores of CAS-R of patients. Note: the abscissa indicated CAS-R, and the ordinate indicated the score. The score of CAS-R of the control group after intervention was (28.74 ± 4.35). The score of CAS-R of the study group after intervention was (31.09 ± 5.12). ^*∗*^indicates the obvious difference in the scores of CAS-R between groups after intervention (*t* = 2.754, *P*=0.007).

**Figure 3:** ROC curve of patients.

**Table 1:** General data.

Observation indexes	Control group (*n* = 62)	Study group (*n* = 62)	*t*/*X*^2^	*P* value
Age (years old)	64.84 ± 6.71	65.19 ± 7.02	0.284	0.777
BMI (kg/m^2^)	22.65 ± 3.41	22.73 ± 3.50	0.129	0.898
Course of disease (years)	3.51 ± 1.08	3.47 ± 1.10	0.204	0.838
Gender			0.130	0.719
Male	32 (51.61)	34 (54.84)		
Female	30 (48.39)	28 (45.16)		
Basic diseases				
Hypertension	27 (43.55)	29 (46.77)	0.130	0.718
Diabetes	35 (56.45)	33 (53.23)	0.130	0.718
Hyperlipemia	32 (51.61)	30 (48.39)	0.129	0.719
High cholesterol	29 (46.77)	26 (41.94)	0.294	0.588
Education degree			0.292	0.589
Middle school degree and above	35 (56.45)	32 (51.61)		
Middle school degree and below	27 (43.55)	30 (48.39)		

**Table 2:** Patients' self-efficacy.

Evaluation dimension	Control group (*n* = 62)	Study group (*n* = 62)	*X* ^2^	*P* value
Regular returning visit	24 (38.71)	51 (82.26)	24.598	<0.001
Emotional control	22 (35.48)	55 (88.71)	37.313	<0.001
Monitoring of blood pressure and blood fat	34 (54.84)	57 (91.94)	21.844	<0.001
Exercise	27 (43.55)	48 (77.42)	14.880	<0.001
Diet control	36 (58.06)	58 (93.55)	21.282	<0.001
Reasonable diet structure	25 (40.32)	49 (79.03)	19.304	<0.001
Timely medication	36 (58.06)	60 (96.77)	26.571	<0.001
Medication conforming to dosage	32 (51.61)	59 (95.16)	30.102	<0.001
Persistent medication	27 (43.55)	55 (88.71)	28.228	<0.001
Quitting smoking	30 (48.39)	51 (82.26)	15.700	<0.001
Quitting drinking	28 (45.16)	46 (74.19)	10.858	<0.001

**Table 3:** Area under curve.

Test result variables	Area	Standarderror^a^	AsymptoticSig.^b^	Asymptotic 95% confidence interval
12-lead Holter ECG combined with mobile Internet + routine ECG	0.976	0.024	0.105	0.000–1.000
12-lead Holter ECG combined with mobile Internet	0.960	0.034	0.117	0.000–1.000
12-lead Holter ECG	0.944	0.044	0.130	0.000–1.000
Routine ECG	0.734	0.162	0.425	0.000–1.000

^a^indicates nonparametric assumptions; ^b^indicates zero hypothesis, real area = 0.5.

## Data Availability

Data used to support the findings of this study are available on reasonable request from the corresponding author.
